This article has been retracted.

# Parallel declines in abundance of insects and insectivorous birds in Denmark over 22 years

**DOI:** 10.1002/ece3.5236

**Published:** 2019-05-15

**Authors:** Anders Pape Møller

**Affiliations:** ^1^ Ecologie Systématique Evolution, Université Paris‐Sud, CNRS, AgroParisTech Université Paris‐Saclay Orsay Cedex France; ^2^ College of Life Sciences Beijing Normal University Beijing China

**Keywords:** agriculture, Diptera, farming practice, insectivorous birds, land use, windscreen

## Abstract

1. Farmers in most western countries have increased use of fertilizer and pesticides with impact on wild animals and plants, including the abundance of insects and their predators.
2. I used 1,375 surveys of insects killed on car windscreens as a measure of insect abundance during 1997–2017 at two transects in Denmark. I cross‐validated this method against three other methods for sampling insect abundance, and I investigated the effects of this measure of insect abundance on the abundance of breeding insectivorous birds.
3. The abundance of flying insects was quantified using a windscreen resulting in reductions of 80% and 97% at two transects of 1.2 km and 25 km, respectively, according to general additive mixed model. Insect abundance increased with time of day, temperature, and June date, but decreased with wind resulting in a reduction by 54%. The abundance of insects killed on a car windscreen was strongly positively correlated with the abundance of insects caught in sweep nets and on sticky plates in the same study areas and at the same time as when insects were sampled using windscreens. The decline in abundance of insects on windscreens predicted the rate at which barn swallows *Hirundo rustica* fed their nestlings, even when controlling statistically for time of day, weather, and age and number of nestlings. The abundance of breeding pairs of three species of aerially insectivorous birds was positively correlated with the abundance of insects killed on windscreens at the same time in the same study area. This suggests a link between two trophic levels as affected by the temporal reduction in the abundance of flying insects.
4. These findings are consistent with recent dramatic declines in insect abundance in Europe and North America with consequences for the rate of food provisioning of barn swallow offspring, the abundance of aerially insectivorous birds and bottom‐up trophic cascades.

## 1 INTRODUCTION

Insects constitute most species (May, 1988), and they hence play important roles as decomposers, pollinators, and herbivores acting as prey for higher trophic levels (Gullan, 1994). A number of studies have recently shown dramatic reductions in the biomass and the abundance of insects (Fox et al., 2014; Hallmann et al., 2017; Vogel, 2017). The abundance of flying insects has been reduced by more than 75% since 1990 even within nature reserves in Germany (Hallmann et al., 2017; Vogel, 2017). Similarly, Fox et al. (2014) reported a decrease of 28% in total moth abundance during 1968–2007 in the UK. These reductions have been attributed to altered agricultural practice and land use. Thus, large declines in the diversity and the abundance of insects during a period of just a few decades must imply dramatic effects on ecosystems (Lister & Garcia, 2018). This time frame is of the highest relevance and the data presented here cover exactly this period of time raising questions about the ultimate causes of such changes.

Climate change has been suggested to affect the phenology and the abundance of ectothermic organisms (Thackeray et al., 2010). Because ecto‐ and endothermic organisms are affected differently by climate change, organisms at different trophic levels are not impacted similarly (Thackeray et al., 2010). Consistent with this suggestion, insect abundance has been closely related to current weather conditions (Kang & Kaller, 2013; Møller, 2001, 2013; Teglhøj, 2017; Turner, 1980). Local insect availability increases with temperature and decreases with wind speed, cloud cover, and precipitation. However, there are also close associations between insect availability and abundance, respectively, and time of day and time during the season with insects emerging earlier than just a few years ago (Møller, 2001, 2013; Taylor, 1974; Turner, 1980).

Humans commonly change the abundance, biodiversity, and food availability for many organisms through effects on agriculture, forestry, aquaculture, and fisheries. Recent studies have shown a reduced abundance of insects associated with the amount and the kind of pesticides used in agriculture (Nocera et al., 2012; Pomfret, Nocera, Kyser, & Reudink, 2000; Poulin, Lefebvre, & Paz, 2010). There have been changes in composition of the diet of insectivores as revealed by the content of dichloro‐diphenyl‐trichloroethane in historical samples of insects exploited by insectivorous birds (Nocera et al., 2012). From a statistical point of view, strong relationships between components of global change may imply collinearity, thereby making it difficult to identify the exact underlying mechanisms responsible for changes in ecosystems and their component parts.

Here, I analyzed a long‐term data set for 1997–2017 on the abundance of insects and the impact of this change in abundance on food availability for aerial insectivorous birds. The objectives of this paper were to (a) quantify the temporal decline in abundance of insects; (b) test for differences in reduction in insect abundance among sampling methods since different sampling methods may differ in their ability to monitor insect abundance; and (c) test for differences in the effects of abundance of insects on predator abundance, that is, insectivorous birds such as swallows and martins. I did so by relying on an extensive study of insect abundance in Denmark during 1997–2017 and the simultaneous abundances of aerially insectivorous birds that rely on flying insects for successful reproduction.

## 2 MATERIAL AND METHODS

### 2.1 Study sites

I studied insects and birds at Kraghede (57°12′N, 10°00′E), Denmark in an open farmland habitat during 1997–2017 (Møller, 1994, 2013). This 45 km^2^ study area consists of scattered farms and houses interspersed by meadows and fields where the main crops are wheat and potatoes. Hedgerows, small plantations, ponds, streams, and ditches are dispersed across the study area. There was little or no change in land use in the study area during 1997–2017 with the kinds of crops and their spatial extent remaining stable (wheat accounted for 45% and potatoes 15% with beets, maize, rye, and other crops being stable). Barn swallows *Hirundo rustica* breed inside barns and houses and rarely under bridges, while house martins *Delichon urbicum* place their nests outside on buildings and sand martins *Riparia riparia* dig tunnels for their nests in sand pits or in the banks of streams.

### 2.2 Insect samples

Flying insects were sampled as the number of insects killed on the windscreen of a car when driven at a fixed speed of 60 km/hr on a specific road (transect) of 1.2 km at Kraghede, Denmark and a second road of 25 km across the study area at Pandrup, Denmark (Møller, 2013; Appendix S1). These data were cross‐validated across alternative methods (Appendices S2 and S3). All surveys of insects were made using rental cars with 2–3 cars being used each year (Appendix S4). These two study sites at Kraghede and Pandrup were separated by 12 km, and while the study site at Kraghede mainly consisted of sandy soil, that at Pandrup mainly consisted of sphagnum. Differences in soil implied that the two study sites differed in crops and domestic husbandry. High abundance of insects is associated with large numbers of insects being smashed on the windscreen of cars (Møller, 2013; Vogel, 2017). Hence, the number of insects on the windscreen provides an estimate of insect abundance (Møller, 2013). The effect of car brand on the abundance of insects killed on the windscreen did not reach statistical significance (Table 1). Likewise, there was no significant interaction. This is not surprising given that 2–3 different rental cars were used for the study. I collected 1,375 insect samples on the 1.2 km transect at Kraghede during 1997–2017 ranging from 44 to 111 per year, with an average of 65.5 samples per year (95% CL 59.9 71.9), *N* = 21 years. In addition, I collected 157 insect samples during 2014–2017 on a 25 km transect at Pandrup. Insects were sampled across the breeding season of the insectivores from May 18 to September 16, mean (*SE*) July 2 (0.70) with one to five samples per day collected from early morning (6:00) to late evening (21:30). Insect counts were significantly repeatable when comparing multiple samples collected the same day relative to the samples collected on different days (repeatability *R* = 0.47 (*SE* = 0.03), *F* = 3.26, *df* = 347, 548, *R* ^2^ = 0.67, *p* < 0.001; Falconer & Mackay, 1996).

**Table 1:** General additive mixed model (GAMM) of insect abundance killed on the windscreen of a car (Gaussian distributed response variable with an identity link function) in relation to year, time of day, temperature, wind, car model, year by car model interaction, June date, and year by June date interaction

Variable	edf	Ref. *df*	*F*	*p*
Year	3.36	4.11	9.844	<0.0001
Time of day	4.26	46.72	13.024	<0.0001
Temperature	6.17	7.71	4.662	<0.0001
Wind	2.70	2.92	39.240	<0.0001
Car model	0.003	7	0.000	0.352
Year × Car model	1.47	7	0.367	0.120
June date	79.30	98	6.817	<0.0001
Year × June date	0.000	98	0.000	0.524

Note

Fixed factors were year, time of day, wind, and temperature, while random effects were car model and June date. Adjusted *R*‐squared was 0.611, and the deviance explained was 65%. edf and Ref. *df* are the degrees of freedom for the smoothing term. The test was based on 1,355 transects.

I used four different methods to assess insect abundance in my study area. First, I recorded the abundance of insects on the windscreen, under the assumption that data obtained with the three additional methods should be strongly positively correlated if they were estimating the same phenomenon. Second, I also recorded insect abundance with sweep‐net samples at the farms where barn swallows were breeding during 1997–2011 at the same time during the day as when insects were recorded using information on the abundance of insects on windscreens. Sweep nets had a shaft of 1 m and a net opening with a diameter of 50 cm. A total of ten sweeps were made with the sweep net while walking at a speed of 5 km/hr across fields at a maximum distance of 100 m from the nearest breeding site. Third, I sampled insects on sticky plates (EcoStyle®) with a surface of 640 cm^2^ during June 10–July 5 2017 by placing two traps within a 100 m radius of each barn swallow nest site since most foraging activities by barn swallows occur <200 m from the nest (Møller, 1994, 2013; Turner, 1980). All insect plates were placed 1.5 m above ground, assuming that this is the most common foraging height for barn swallows (Bryant & Turner, 1982; Kang & Kaller, 2013; Møller, 1994; Teglhøj, 2017). The two individual insect sampling stations per nest allowed for statistical test of repeatability. Fourth, I recorded the rate at which adult barn swallows fed their nestlings (feeding rate). To determine whether there was a significant effect of insect abundance on feeding rate, I conducted the plate samples during the same time that insects were being collected on the windscreen. It is known that when there are more insects, barn swallows feed their offspring at a higher rate than when insects are rare (Møller, 1994; Turner, 1980). To further analyze this pattern, I obtained records of temperature, wind speed, and precipitation daily at the same exact study site during each feeding rate record.

### 2.3 Insects, feeding rate of nestling barn swallows and abundance of insectivores

I searched all suitable breeding sites of the three species of hirundines at weekly intervals during 1971–2017 within the same 45 km^2^ study area using a similar extent of search effort. I located nests of barn swallows inside farm buildings, nests of house martins under the eaves of outside buildings and nests of sand martins in the small number of sand pits and tunnels dug out in the banks of streams.

Both adult barn swallows attending a nest provide nestlings with food. Feeding rate was recorded as the number of times male and female nest owners fed their offspring during daily observation periods of 1 hr. Such feeding rates per hour are highly repeatable within and among days (Møller, 1994), thus providing reliable information. I recorded the rate at which parent barn swallows fed their nestlings (feeding rate) during one‐hour observation periods twice for 149 nests during May–August 1997–2017. Feeding rates were recorded on the same dates and immediately before or after insect samples were collected using car transects.

### 2.4 Statistical analyses

I used a general additive mixed model (GAMM; van Rij, 2015) to test for a relationship between insect abundance with a Gaussian distribution and an identity link function and year, time, temperature, car model, year by car model interaction, June date, and year by June date interaction. GAMM was used to account for the fact that data such as insect abundance in this study show temporal auto‐correlation.

I tested if insect abundance as assessed by insects killed on the windscreen was consistent between 1.2 and 25 km transects using a GLM model with insect abundance as a Poisson distributed response variable with a log link function. There was no significant overdispersion in these tests.

I used two GLM models with insect abundance as a Poisson distributed response variable and a log link function to test whether the abundance of insects killed on the windscreen was positively related to the number of insects caught with a sweep net and the abundance of insects on sticky plates, respectively.

I tested in a GLM using feeding rates as a log‐transformed response variable with an identity link function and nest identity, the abundance of insects, brood size, age of nestlings, time of day, time of day squared, air temperature, wind speed, and cloud cover as predictor variables. I analyzed in a GLM whether the abundance of insects as a response variable that was Poisson distributed with a log link function could be related to year, date, time of day, cloud cover, wind, and temperature, with time squared included to account for any curvilinear relationship during the day.

I tested in a GLM whether the abundance of insects as a Poisson distributed response variable with a log link function was positively related to weather conditions. Furthermore, I tested in a GLM whether insect abundance on the windscreen as a response variable that was Poisson distributed with a log link function was related to year, date, date squared*year, time, time squared, wind, cloud cover, and temperature as predictor variables. I also tested whether mean annual abundance of insects in a GLM model that included the number of insect counts per year declined over time.

I tested in a GLM whether the number of feeds per barn swallow nestling and per hour as a Poisson distributed variable and a log link function increased with the abundance of insects recorded on the windscreen. Furthermore, I tested in a GLM with Poisson distributed data and a log link function whether the abundance of insects on the windscreen was affected by June date, time, temperature, wind, age of nestlings (days), and number of nestlings. I also tested in a GLM with Poisson distributed data and a log link function whether the abundance of three hirundine species increased with the abundance of insects on the windscreen.

I calculated variance inflation factors (VIF) to estimate problems of collinearity, but maximum VIF was always <2.5, implying weak collinearity (McClave & Sincich, 2003). All analyses were made with JMP (SAS, 2012) except for the GAMM, which was made using R Core and Team (2016).

## 3 RESULTS

A GAMM accounted for almost 61% of the variance in the abundance of insects (Table 1). Insect abundance based on insects killed on the windscreen decreased by 80% during 1997–2017 for the 1.2 km transect according to the GAMM (Figure 1, Table 1). Closer inspection of the temporal trend and the overlap in confidence intervals revealed a relatively stable trend between the years 1997 and 2010 with a significant decline during 2010–2017 (Figure 1). There were additional significant effects of time of day (insect abundance increasing during the day), temperature (insect abundance increased with temperature), wind (insect abundance decreased with wind) and June date (insect abundance increasing during the summer) (Table 1). All weather variables were recorded following each insect survey. In contrast, there was no significant effect of car model (Table 1) and year by June date interaction (Table 1), while there was a weak, but significant year by car model interaction (Table 1).

**Figure 1:** The residual number of insects from a general additive mixed model at Kraghede, Denmark during 1997–2017 after controlling for the variables listed in Table 1. The line is the regression line and the band is the 95% confidence interval

The abundance of insects changed in relation to (2A) temperature, (2B) time of day, and (2C) the interaction between temperature and time of day.

The abundance of three species of insectivorous birds belonging to the family Hirundinidae increased with the number of insects killed on the windscreen (Figure 3; Table 2). The size of the breeding population of barn swallows, house martins, and sand martins decreased significantly during 1997–2017 (3A, barn swallow: GLM with Poisson distributed data and a log link function; *χ* ^2^ = 164.25, *df* = 1, *p* < 0.0001, 95% CL −0.036, −0.027; 3B, house martin: *χ* ^2^ = 27.03, *df* = 1, *p* < 0.0001, 95% CL −0.075, −0.034; 3C, sand martin: *χ* ^2^ = 21.28, *df* = 1, *p* < 0.0001, 95% CL −0.057, −0.023). Inspection of the relationships revealed strongly increasing population sizes of swallows and martins at high abundance of insects (Figure 2).

**Table 2:** Abundance of barn swallows, house martins, and sand martins in relation to the number of insects killed on the windscreen during 1997–2017

	LR *χ* ^2^	*p*	Lower 95% CL	Upper 95% CL	Increase
Barn swallow	20.63	<0.0001	0.176	0.441	+32%
House martin	13.11	0.0003	0.354	1.180	+100%
Sand martin	60.36	<0.0001	1.044	1.746	+254%

Note

GLMs show large declines in bird abundance. LR is likelihood‐ratio *χ* ^2^. Sample sizes were 20 in each analysis.

**Figure 2:** The number of insects from a GLM at Kraghede, Denmark during 1997–2017 in relation to (a) temperature (°C), (b) time of day, and (c) temperature by time of day interaction

**Figure 3:** The number of breeding pairs of (a) barn swallow, (b) house martin, and (c) sand martin at Kraghede, Denmark, in relation to the number of insects killed on the windscreen of a car. The lines are the regression lines and the bands around estimates are 95% confidence intervals

## 4 DISCUSSION

The abundance of flying insects in a farmland area in Denmark as revealed by numbers killed on the windscreen of a car decreased by more than 80% during 1997–2017. Declines in insect abundance were consistent across sites, sampling methods (insects killed on the windscreen, sweep nets, sticky traps, and feeding rates) and change in climate conditions. The rate at which adult barn swallows fed their nestlings (feeding rate) was strongly positively correlated with the abundance of insects on windscreens recorded at the same time as insects on the windscreen, and higher abundance of insects also implied higher abundance of three species of aerially insectivorous birds, suggesting that the measure of insect abundance on cars was biologically relevant for birds consuming insects.

Insects are commonly killed on the windscreen of cars, although this has generally been considered a nuisance rather than a biologically relevant measure of insect abundance. Here, I validated the measure of insect abundance from car windscreens. I used insects killed on windscreens, sweep‐net captures, sticky plates, and feeding rates by barn swallows to obtain four independent measures of insect abundance, showing consistent estimates of insect abundance among methods.

Declines in insect abundance and biomass on farmland estimated from transects with cars are high. Shortall et al. (2009) and Hallmann et al. (2017) documented declines in insect biomass reaching 75% during a period of 27 years. Declines in insect abundance may have a number of causes including altered land use, novel pesticides, climate warming, and invasive predators. Previously published effects of climate on abundance of insects are partly due to advanced phenology of insects (Both, 2010; Both et al., 2010; Visser, 2008). Hence, I included ambient temperature in the statistical models because it had changed considerably in the study area since 1997. However, the relative decline in insect abundance during 1997–2017 still reached 54% after controlling statistically for the partial effects of changing climate (temperature and wind). While heatwaves may compromise sperm function and cause transgenerational damage (Sales et al., 2018), we should expect the opposite result of what I found here. Therefore, reductions in insect abundance must be attributed to other factors such as agricultural practice or pesticide use.

The abundance of insects on the windscreen of a car is a biologically relevant estimate of food availability for barn swallows. Indeed, the rate at which barn swallows fed their young is strongly positively correlated with the abundance of insects on the windscreen of a car, even when controlling statistically for potentially confounding variables such as changing weather conditions. Furthermore, population size of barn swallows, house martins, and sand martins was strongly positively correlated with the abundance of insects on windscreens. Therefore, insect abundance estimated from the number of insects killed on a windscreen is biologically relevant for insectivorous birds.

The findings reported here may have important implications. There are few long‐term studies of insects (Taylor, 1974 is an exception). A number of studies of insects have suggested population declines by more than 75% in recent decades (Hallmann, Foppen, Turnhout, Kroon, & Jongejans, 2014; Hallmann et al., 2017; Nebel, Mills, McCracken, & Taylor, 2010; Nocera et al., 2012; Pomfret et al., 2000; Vogel, 2017). Studies of arthropod abundance in the tropics have precipitated a trophic bottom‐up cascade with effects on lizards, frogs, and birds (Lister & Garcia, 2018). It is important to verify these findings across temporal and spatial scales. It is also important to consider whether alternative measures of insect abundance such as temporal and spatial trends in use of windscreen detergent may represent indirect estimates of insect abundance. Similarly, the amount of pesticides used in agriculture may reduce insect abundance. Finally, the spatial and temporal use of mosquito spray should reflect the spatial and temporal patterns of abundance of mosquitoes and other biting insects.

## 5 CONCLUSIONS

This 21‐year study of insect abundance showed a tenfold decline. The decline in insect abundance reported here could partly be attributed to changes in climate. Such declines in insect abundance may have consequences for reproductive success in insectivorous birds such as hirundines, but also have consequences for population size as documented in the present study. Long‐term population declines in abundance of insects must have important consequences for insectivores, interspecific interactions, and ecosystem functioning.

## CONFLICT OF INTEREST

The author declares no conflict of interest.

## AUTHOR CONTRIBUTIONS

APM developed the idea, collected and analyzed the data and wrote the paper.

## Data Availability

All data are available at https://doi.org/10.5061/dryad.gq73493.
